The article "Abdominal Pseudocyst: A Rare Complication of Ventriculoperitoneal Shunts" was retracted in 2024. Reasons: false authorship; unreliable results or conclusions; no approval from an author; concerns about the authorship.

# Abdominal Pseudocyst: A Rare Complication of Ventriculoperitoneal Shunts

**DOI:** 10.7759/cureus.18956

**Published:** 2021-10-21

**Authors:** Turki M Bin Saqyan, Lama I Basunbul, Ahmed A Badahdah, Yasir A Saleh, Suhail S Filimban, Ali A Alwabari, Ahmad A Almutairi, Sultanah R Alanazi, Abdulrazaq S Alghamdi, Bader O Aldadi, Bakheet A Alghamdi, Shafi A Alzahrani, Ahmed R Alzahrani, Osama H Alghamdi, Malak Alshammari

**Affiliations:** 1 College of Medicine, Prince Sattam Bin Abdulaziz University, Al-Kharj, SAU; 2 College of Medicine, King Abdulaziz University, Jeddah, SAU; 3 College of Medicine, King Saud University, Riyadh, SAU; 4 College of Medicine, Umm Al Qura University, Mecca, SAU; 5 College of Medicine, Vision Colleges, Riyadh, SAU; 6 College of Medicine, Northern Border University, Arar, SAU; 7 College of Medicine, Al-Baha University, Al-Baha, SAU; 8 College of Medicine, Imam Abdulrahman Bin Faisal University, Dammam, SAU

**Keywords:** case report, gait ataxia, ventriculoperitoneal shunt, abdominal mass, normal pressure hydrocephalus

## Abstract

We present the case of a 69-year-old man patient who was brought with a history of gait disturbances, memory impairment, and urinary incontinence with gradual worsening over the past six months. The patient underwent magnetic resonance imaging of the brain which demonstrated enlarged ventricles, widening of the Sylvian fissure, and narrow sulci at the vertex. Subsequently, the patient underwent a lumbar puncture which revealed a normal opening pressure with normal cerebrospinal fluid analysis. The diagnosis of normal pressure hydrocephalus was established. The patient underwent a ventriculoperitoneal shunt for the management of his symptoms. Three years after the placement of the shunt, the patient was brought to the emergency department with an expanding right-sided subcutaneous abdominal mass. A computed tomography scan of the abdomen showed the subcutaneous mass superficial to the right rectus muscle and was containing the coiled distal end of the shunt. Such findings were consistent with a subcutaneous cerebrospinal fluid pseudocyst. The mass was aspirated and the fluid analysis was in keeping with the cerebrospinal fluid characteristics. The fluid culture revealed no bacterial growth. The ventriculoperitoneal shunt was replaced with a minimally invasive technique.

## Introduction

Normal-pressure hydrocephalus is a potentially reversible disorder that is characterized by the triad of cognitive impairment, urinary urgency or incontinence, and gait disturbances [1]. It is the most frequent cause of hydrocephalus in adults. The idiopathic normal pressure hydrocephalus is a disorder of the elderly with an average age of onset at 70 years. The disorder does not have any sex predilection. The exact pathophysiology of this disorder remains unclear. However, several explanations have been suggested. Examples of such explanations include the hyperdynamic flow of the cerebrospinal fluid and impairment in the fluid reabsorption [2]. While the diagnosis of normal pressure hydrocephalus is suggested by its clinical features, supportive assessment by magnetic resonance imaging and cerebrospinal fluid drainage may be required for confirming the diagnosis. The ventriculoperitoneal shunt is used for the management of this disorder and results in improvement [3]. Here, we present the case of an elderly patient with normal pressure hydrocephalus who underwent a ventriculoperitoneal shunt. The patient developed a subcutaneous cerebrospinal fluid pseudocyst, a very rare complication of shunts.

## Case presentation

We present the case of a 69-year-old male patient who was brought to the outpatient clinic by his daughter as he developed gait disturbances, memory impairment, and urinary incontinence with gradual worsening over the past six months. He reported having a history of falls because of his unbalanced gait. The patient started to have difficulty with findings words and had problems with concentration. There was no history of headache, muscle weakness, hallucination, or changes of personality. The past medical history of the patient was remarkable for long-standing hypertension, diabetes mellitus, and dyslipidemia. His surgical history is remarkable for inguinal hernia repair and appendectomy. The patient is retired and lives with his daughter.

On physical examination, the vital signs were within the normal limits. The neurological examination revealed decreased attention span and impaired concentration. However, the patient had normal fluency and normal naming of objects. The muscle tone, power, and coordination were normal in both the upper and lower limbs. Gait examination showed normal posture and speed but was wide-based. Cranial nerves examination was normal. Initial laboratory findings were within the normal limits (Table 1). The Mini-Mental State Examination revealed mild cognitive impairment with a score of 27 out of 30. The patient underwent magnetic resonance imaging of the brain which demonstrated enlarged ventricles, widening of the Sylvian fissure, and narrow sulci at the vertex (Figure 1). The clinical and radiological findings were suggestive of the diagnosis of normal pressure hydrocephalus. Subsequently, the patient underwent a lumbar puncture which revealed a normal opening pressure with normal cerebrospinal fluid analysis. The patient underwent a ventriculoperitoneal shunt for the management of the normal pressure hydrocephalus. One year after the placement of the shunt, the patient demonstrated a marked improvement in his gait and resolution of urinary incontinence.

**Table 1:** Summary of the results of laboratory findings

Laboratory Investigation	Unit	Result	Reference Range
Hemoglobin	g/dL	14.2	13.0–18.0
White Blood Cell	1000/mL	7.5	4.0–11.0
Platelet	1000/mL	350	140–450
Erythrocyte Sedimentation Rate	mm/hr.	14	0–20
C-Reactive Protein	mg/dL	7.2	0.3–10.0
Total Bilirubin	mg/dL	0.9	0.2–1.2
Albumin	g/dL	4.2	3.4–5.0
Alkaline Phosphatase	U/L	53	46–116
Gamma-glutamyltransferase	U/L	47	15–85
Alanine Transferase	U/L	58	14–63
Aspartate Transferase	U/L	25	15–37
Blood Urea Nitrogen	mg/dL	16	7–18
Creatinine	mg/dL	1.1	0.7–1.3
Sodium	mEq/L	135	136–145
Potassium	mEq/L	3.9	3.5–5.1
Chloride	mEq/L	105	98–107

**Figure 1:** Magnetic Resonance Imaging Magnetic resonance T2-weighted image demonstrated enlarged ventricles, widening of the Sylvian fissure, and narrow sulci at the vertex.

Three years after the placement of the shunt, the patient was brought to the emergency department with an expanding right-sided subcutaneous abdominal mass. The mass was soft and has a smooth surface with normal overlying skin. Ultrasound examination of the abdominal wall revealed a well-defined anechoic with fluid density measuring approximately 7 x 5 x 6 cm. The differential diagnosis for this mass was an abscess, lymphocyte, seroma, and cerebrospinal fluid. A computed tomography scan of the abdomen showed the subcutaneous mass superficial to the right rectus muscle and was containing the coiled distal end of the shunt (Figure 2). Such findings were consistent with a subcutaneous cerebrospinal fluid pseudocyst. The mass was aspirated and the fluid analysis was in keeping with the cerebrospinal fluid characteristics. The fluid culture revealed no bacterial growth. The ventriculoperitoneal shunt was replaced with a minimally invasive technique.

**Figure 2:** Computed Tomography Images Selected computed tomography images in the axial (A) and coronal (B) planes demonstrating a fluid-filled subcutaneous lesion (arrow) adjacent to the right abdominal rectus muscle with hyperdensities located at the periphery of the lesion which is the coiled distal end of the shunt.

## Discussion

We presented the case of a patient with normal pressure hydrocephalus who was managed with ventriculoperitoneal shunt and developed a cerebrospinal fluid pseudocyst in the subcutaneous tissue, which is a very rare complication. Diversion of the cerebrospinal fluid flow through shunt placement is the most common neurosurgical procedure. The shunt can result in significant benefits to patients. However, this procedure is not without any complications [4].

Desai et al. [5] conducted a retrospective study involving 476 patients with a ventriculoperitoneal shunt in a single institution for five years duration. The study revealed that the overall complication rate of the shunt was 19%. The complications included infection, shunt failure, subdural hematoma, and other shunt-related complications [6]. Generally, the most complication of shunts is overdrainage. In contrast, pseudocyst is among the rare complications of shunts. The clinical manifestation of pseudocyst includes abdominal pain with swelling. However, children tend to develop neurological symptoms more commonly [7].

The cerebrospinal fluid pseudocyst is primarily diagnosed based on the detailed medical history and the physician needs to have a high index of suspicion for this complication. The time interval between the placement of the ventriculoperitoneal shunt and the development of pseudocyst varies from a few weeks to several years [8]. The pseudocyst typically develops in the peritoneal cavity [9]. The peritoneal pseudocyst may be managed by laparoscopic or laparotomy approaches [10]. The development of the pseudocyst in the subcutaneous tissue, as in our case, is very unusual.

## Conclusions

The cerebrospinal fluid pseudocyst is a very rare complication of ventriculoperitoneal shunt placement. The pseudocyst may develop in the subcutaneous tissue. Clinicians should be aware of this complication and maintain a high index of suspicion for pseudocyst when they encounter a patient with a shunt presenting with abdominal swelling. The diagnosis can be readily made by computed tomography scan.
